The article "Application of Deep Learning for Early Screening of Colorectal Precancerous Lesions under White Light Endoscopy" was published in 2020. Journal: Comput Math Methods Med.

# Application of Deep Learning for Early Screening of Colorectal Precancerous Lesions under White Light Endoscopy

**DOI:** 10.1155/2020/8374317

**Published:** 2020-08-18

**Authors:** Junbo Gao, Yuanhao Guo, Yingxue Sun, Guoqiang Qu

**Affiliations:** ^1^Information Engineering College, Shanghai Maritime University, Shanghai 201306, China; ^2^Department of Gastroenterology, Eastern Hospital, Shanghai Sixth People Hospital, Shanghai 201306, China

## Abstract

**Methods:**

We collected and sorted out the white light endoscopic images of some patients undergoing colonoscopy. The convolutional neural network model is used to detect whether the image contains lesions: CRC, colorectal adenoma (CRA), and colorectal polyps. The accuracy, sensitivity, and specificity rates are used as indicators to evaluate the model. Then, the instance segmentation model is used to locate and classify the lesions on the images containing lesions, and mAP (mean average precision), AP_50_, and AP_75_ are used to evaluate the performance of an instance segmentation model.

**Results:**

In the process of detecting whether the image contains lesions, we compared ResNet50 with the other four models, that is, AlexNet, VGG19, ResNet18, and GoogLeNet. The result is that ResNet50 performs better than several other models. It scored an accuracy of 93.0%, a sensitivity of 94.3%, and a specificity of 90.6%. In the process of localization and classification of the lesion in images containing lesions by Mask R-CNN, its mAP, AP_50_, and AP_75_ were 0.676, 0.903, and 0.833, respectively.

**Conclusion:**

We developed and compared five models for the detection of lesions in white light endoscopic images. ResNet50 showed the optimal performance, and Mask R-CNN model could be used to locate and classify lesions in images containing lesions.

## 1. Introduction

Colorectal cancer (CRC) is a common malignancy of the digestive system. According to the latest data, the morbidity and mortality of CRC rank among the top four in cancer [1]. With the improvement of Chinese people's living standards, the incidence of CRC increases year by year. The most common precancer disease of CRC is colorectal adenoma (CRA) [2]. At present, total colonoscopy is still the best screening method for colorectal polyps, CRA, and CRC [3]. Early detection of CRA and endoscopic resection of adenoma under colonoscopy can reduce or avoid the occurrence of CRC, thereby reducing the mortality rate of CRC [4, 5]. Early diagnosis of digestive system tumours has always been a hot spot for the medical community to conquer. However, it is difficult to detect early precancerous lesions of the digestive system because they generally involve a small range and are shallow in depth, and the morphological manifestations under endoscopy are not obvious [6]. Moreover, the evaluation results of endoscopy often depend on the subjective experience of the operating physician, which is highly subjective and requires a high level of clinical skills and work experience of the physician. The low-qualified or fatigued physician is more likely to misdiagnose the lesion [7].

At present, the application of artificial intelligence (AI) in the medical field has shown an exciting dawn, and its exploration in the field of digestive endoscopy has also achieved some preliminary results [8]. In the study conducted by [9], two different shape description features were compared to distinguish whether there are polyps in the colorectal region. The algorithm was tested on 300 images, among which 150 images contain polyps and 150 images of normal mucosa, with an accuracy of 86%. In the study [10], the author used the fitting ellipse method and multiscale Gaussian texture geometric features, and the true positive of the algorithm was 64.8%. Reference [11] combined the advantages of wavelet transform and local uniform binary mode to characterize image features and used support vector machine (SVM) as the classifier. Their data set contained a total of 1200 images (600 polyp images and 600 nonpolyp tissue images), and the algorithm accuracy reached 91.6%.

With the emergence of deep learning algorithm, machine learning has gradually gotten rid of the limitation of low efficiency and imprecision in manually extracting data features, which has brought revolutionary progress to the research and development of artificial intelligence. Zhang et al. [12] used white light endoscopic images to distinguish polyps from adenoma, with an accuracy rate of 85.9%. Patino-Barrientos et al. [13] used the VGG16 model to perform Kudo's Classification for Colon Polyps on white light endoscopic images. The accuracy rate was 83%, and the F1 score was 0.83. Ruikai et al. [14] used the YOLOv3 algorithm to detect and locate polyps on white light endoscopes. The accuracy of the results was 88.6%, and the recall rate was 71.6%.

In summary of the above studies, it can be concluded that the application of convolutional neural network of deep learning in the detection, location, and classification of colorectal polyps is feasible and has achieved good results. Moreover, due to the late development of endoscopic medical technology in China, the overall technical level lags behind that of developed countries, so most of the endoscopic techniques used in hospitals in China are still dominated by ordinary white light endoscopes. In the daily diagnosis, the endoscopist must thoroughly examine each image of each patient; the process is very cumbersome. Therefore, the development of a computer-aided diagnosis system based on white light endoscopy can greatly reduce the burden on medical personnel and is of great significance.

The contribution of our study is to establish a model of detection, localization, and classification of colorectal lesions based on white light endoscopy. Compared with other models based on the research of white light endoscopy, the models of this study have improved to some extent in some evaluation indicators of experimental results. In the process of detecting whether white light endoscopic pictures contain lesions, we compared five convolutional neural network models. As a result, the ResNet50 model showed higher detection performance; it scored an accuracy of 93.0%, a sensitivity of 94.3%, and a specificity of 90.6%. In the process of locating and classifying lesions, the Mask R-CNN model was used to segment the images, and a satisfactory result was obtained; its mAP, AP_50_, and AP_75_ were 0.676, 0.903, and 0.833, respectively.

## 2. Materials and Method

### 2.1. Data Set

In this study, images of patients undergoing colorectal examination under white light endoscopy (as shown in Figure 1) were used.

These images were derived from the Digestive Endoscopy Centre, East Hospital, Shanghai Sixth People's Hospital, China. The time span is from June 2015 to September 2019. We created a database containing 3413 WLE images of dimensions 420 × 389 × 3 (RGB), of which 1709 of them contained lesions (CRC, CRA, and polyps) and 1704 of them are normal colorectal mucosa. Images with clear surface and boundary under the white light endoscope and complete film were selected, and corresponding microscope pathology was recorded, which was marked and classified by trained endoscopy physicians and gastroenterologists. Images of normal mucosa have varying degrees of cleanliness and air bubbles. All images containing lesions have been checked to ensure the accuracy of the data set. We randomly divide the image into a training set, a validation set, and a test set (respectively, 70%, 15%, and 15% of the full data set), and limit the balance between the validation set and the test set.

### 2.2. Study Design

In this study, we will follow the following process (Figure 2) to detect, locate, and classify white light endoscopic colorectal lesions.

First of all, we will use the convolutional neural network (CNN) [15] model to distinguish whether the white light endoscopic images contain lesions (CRC, CRA, and polyps) and whether output images also contain lesions. Next, an instance segmentation [16] model Mask R-CNN is used on the image containing a lesion to locate the position of the lesion, and a prediction of the corresponding category of the lesion is given.

### 2.3. CNN Architecture

Convolutional neural networks (CNN) are a kind of Feedforward Neural Network that contains convolutional computation and has a deep structure and is one of the representative algorithms of deep learning [17, 18]. LeCun and his collaborators constructed the convolutional neural network LeNet-5 and achieved success in the recognition of handwritten digits [19]. LeNet-5 and its subsequent variants define the basic structure of modern convolutional neural networks. The alternating convolutional layer and pooling layer in its construction are considered to be able to extract the higher-order features of the input image.

We evaluated five network architectures: AlexNet [20], GoogLeNet [21], ResNet50 [22], ResNet18 [23], and VGG19 [24]. These networks all use a hierarchical structure, with the output of the previous layer as the input of the next layer, continuously extracting and building the higher-order features of the input picture. Because our white light endoscopy image data set is not far enough to support from scratch or train the network, we will use transfer learning to use the above-mentioned pretrained CNN convolutional layer as a feature extractor. These pretrained networks use a large amount of image data (including 1000 categories) for training, and on ILSVRC (ImageNet Large-Scale Visual Recognition Challenge) good results have been achieved, so these networks have the ability to classify various images. According to the use of the feature extraction scheme and transfer learning to solve the new classification problem, the last layer or the last three layers of CNN must be fine-tuned. In this study, we changed the final classification layer to output two categories, namely, normal images and images containing lesions.

For the binary classification, the success of classification of WLE images using CNN is measured by accuracy, sensitivity, and specificity, which are widely employed by colleagues to assess the performance of classification. Here is their definition:

(1) $$\begin{array}{c} \text{Accuracy}=\frac{\text{Number of correct predictions}}{\text{Number of positives}+\text{number of negatives}}, \end{array}$$

(2) $$\begin{array}{c} \text{Sensitivity}=\frac{\text{Number of correct positive predictions}}{\text{Number of positives}}, \end{array}$$

(3) $$\begin{array}{c} \text{Specificity}=\frac{\text{Number of correct negaive predictions}}{\text{ Number of negatives}}. \end{array}$$

In this study, we observed that pretrained ResNet50 usually performs better than the other four networks (Table 1). Therefore, we will introduce this network architecture in detail. ResNet50's network consists of 50 layers, including 17 layers (16 convolutional layers and 1 fully connected layer) of learnable weights. Each convolutional layer contains 64 to 2048 kernels of size 1 × 1 and 3 × 3. In order to enhance the robustness of the internal deformation of the class and avoid overfitting, the convolution kernel with a size of 1 × 1 before the shortcut uses the Rectified Linear Unit (ReLU). ReLU, as the activation function of the neural network, defines the nonlinear output of the neuron after linear transformation; here is the definition:

(4) $$\begin{array}{c} f\left(x\right)=\max\left(0,w^{T}x+b\right). \end{array}$$

In order to improve network performance, we have further optimized the network architecture. And the stochastic gradient descent with momentum (SGDM) is used as the optimization algorithm. The learning rate was initially set to 1*e*-4 and was adaptively modified during the training process until the verification criteria were met. The maximum epoch size of the training process is 50. In order to standardize the model and reduce overfitting, image data enhancement is used in the model training process, including rotation, cropping, and mirror conversion. These data enhancement operations do not affect the content or size of the image. Finally, in order to overcome the generalization gap while taking into account the limited GPU memory, a mini batch size of 16 was chosen.

### 2.4. Mask R-CNN Network Architecture

Mask R-CNN was extended from Faster R-CNN [25]. Faster R-CNN is a popular target detection framework, which was extended to the instance segmentation framework by Mask R-CNN. Mask R-CNN [26] is a two-stage framework. The first stage scans the images and relies on the Region Proposal Network (RPN) algorithm [27] to generate proposals (region of interest, or ROI), and the second stage classifies the proposals and generates bounding boxes and masks. Mask R-CNN can effectively detect the target in the image, add a parallel branch for predicting the target mask on its existing branch for border box recognition, and generate a high-quality segmentation mask for each instance. So it was called Mask R-CNN.

Mask R-CNN was trained in the following steps (Figure 3):

**Step 1 .**

Enter an image you want to process and then carry out the corresponding pre-processing operation or the preprocessed picture.

**Step 2 .**

Input it into a pretrained neural network (ResNe50, etc.) to obtain the corresponding feature map.

**Step 3 .**

Set a predetermined ROI for each point in the feature map, so as to obtain multiple candidate ROI.

**Step 4 .**

Send these candidate ROIs into the RPN network for binary classification (foreground or background) and BB regression and filter out some candidate ROIs.

**Step 5 .**

Perform ROI align operation on the remaining ROIs, that is, match the original image with the pixel of the feature map first and then match the feature map with the fixed feature.

**Step 6 .**

Perform operations on each ROI in Fully Convolutional Networks (FCN) for classification, bounding-box regression, and mask generation.

To develop our Mask R-CNN, we selected 1709 images containing lesions (CRC, CRA, and polyps) as the image database. Next, manually label these images to mark the location and correspondence of the lesions in the picture category, which is a tedious labelling task, and finally, we created an image database in MSCOCO format for lesion location and classification. Each image contains a bounding box around the large intestine lesion in the format of [*x*, *y*, width, and height], which specifies the lesion's position and size in the upper left corner of the image. We further divided the images into 70% for training, 15% for validation, and 15% (256 images) for testing the Mask R-CNN network.

In the Mask R-CNN developed in this study, ResNet50 was used as the backbone network. The minimum batch is set to 1, so that each iteration processes multiple image areas from one training image. Each image is controlled by two different parameters, positive training samples and negative training samples. These two values are set to overlap with ground truth boxes by a factor of [0.6-1.0] and [0-0.3], respectively. Considering the bounding box as a true positive box containing lesions, we chose a threshold of 0.7 for the IoU measure, which is a good threshold for calculating the “intersection” of various bounding boxes.

IoU (Intersection-over-Union) represents the overlap rate between the generated candidate bound and the ground truth bound, that is, the ratio of their intersection and union.

(5) $$\begin{array}{c} \text{IoU}=\frac{\text{area }\left(C\right)⋂\text{a}\text{rea }\left(G\right)}{\text{area }\left(C\right)⋃\text{a}\text{rea }\left(G\right)}. \end{array}$$

In this study, we used some outcome indicators that evaluated the MSCOCO data set to evaluate our model, such as mAP (mean average precision), AP_50_, and AP_75_, as the main evaluation criteria for the results.

For the binary classification, the sample can be divided into four cases of true positive (TP), false positive (FP), true negative (TN), and false negative (FN). Precision predicts the correct value in the case of predicting positive samples; recall predicts the correct value in instances with positive labels.

(6) $$\begin{array}{c} \text{Precision}=\frac{\text{TP}}{\text{TP}+\text{FP}}, \end{array}$$

(7) $$\begin{array}{c} \text{Recall}=\frac{\text{TP}}{\text{TP}+\text{FN}}, \end{array}$$

(8) $$\begin{array}{c} \text{mAP}=\int_{0}^{1}P\left(R\right)dR. \end{array}$$

In formula (8), *P* represents precision and *R* represents recall. mAP is the average AP value of multiple verification set individuals. So the higher the mAP score is, the higher the confidence in the test results will be and the more likely polyps will be contained in the boundary box.

## 3. Results and Discussion

### 3.1. Performance of CNN Model

Table 1 lists the performance of different networks after transfer learning in the process of detecting whether white light endoscopic pictures contain lesions, mainly reflected in the accuracy, sensitivity, and specificity of the network. We found that the modified ResNet50 performed significantly better than the other four networks.

The reason why high sensitivity is very important is because the consequences of false negatives (missed polyps) are much more serious than false positives (misdiagnosed as polyps).  Figure 4 shows some examples of misclassified images. Missed polyps (false negatives) and normal mucosa are misidentified as polyps (false positives).

We have observed a situation that easily leads to missed diagnosis of polyps, that is, the size of polyps is small. Usually in endoscopic detection, some smaller polyps are also easily missed [28], but these polyps are less likely to form tumours at advanced stages, and our models are often correct when detecting large polyps, so to a certain extent, the consequences of missed diagnosis of small polyps are reduced.

### 3.2. Performance of Mask R-CNN Model

Since the data set we marked is in MSCOCO format, a series of result metrics of the MSCOCO data set will be used to evaluate our data set. Here is their definition:

mean average precision (AP):

AP: AP at IoU = 0.50 : 0.05 : 0.95 (primary challenge metric),

AP_50_: AP at IoU = 0.50,

AP_75_: AP at IoU = 0.75,

AP_S_: AP for small objects: area < 32^2^,

AP_M_: AP for medium objects: 32^2^ < area < 96^2^,

AP_L_: AP for large objects: area > 96^2^.

Average recall (AR):

AR: AR given 1 detection per image,

AR_10_: AR given 10 detections per image,

AR_100_: AR given 100 detections per image,

AR_S_: AR for small objects: area < 32^2^,

AR_M_: AR for medium objects: 32^2^ < area < 96^2^,

AR_L_: AR for large objects: area > 96^2^.

The results are shown in Table 2.

An example of the Mask R-CNN we developed to locate and classify lesions is presented in Figure 5.

## 4. Conclusions

Due to the late development of endoscopic medical technology in China, the overall technical level lags behind that of developed countries; ordinary white light endoscopy is still the endoscopic technique used in most hospitals in China. The endoscopist needs to examine each image of each patient carefully. The process is cumbersome. Therefore, the development of a computer-aided diagnosis system based on a white light endoscope is of great significance. Compared with other models based on white light endoscopic research, the model developed in this study has improved the effect and can assist the endoscopist in daily diagnosis, which will greatly reduce the daily burden of medical staff.

In this study, we used white light endoscopic images as a screening tool for colorectal lesions. Through comprehensive evaluation of supervised machine learning algorithms, we find that different algorithms have different prediction performances on image data. By comparing the predictive performance of the classifier, we found that ResNet50 is a good model.

In addition, we also annotated images containing lesions, constructed a data set in MSCOCO format, and used the instance segmentation algorithm Mask R-CNN to perform experiments on this data set. Through comparison and analysis of some result indicators, we found that location and classification of colorectal lesions have achieved a good result.

We hope to develop a computer-aided diagnosis system; the process is shown in Figure 6.

Through the combination of the two models, a white light endoscopic image is inputted, the ResNet50 model is used to determine whether it contains a lesion, and the image containing the lesion is then input into the Mask R-CNN model to locate and classify the lesion.

Future work includes exploring architectures such as capsule networks and attention model, which may be difficult to implement but can provide more specific interpretability. Our goal is to develop a more accurate, real-time colorectal lesion detection, localization, and classification model and deploy it on a system where white light endoscopy works to help physicians better perform colonoscopy for patients.

## Figures and Tables

**Figure 1:** Colorectal polyps in different stages of neoplasia and different grades of bowel cleanliness under white light endoscopy.

**Figure 2:** Colorectal lesion detection localization and classification process.

**Figure 3:** Mask R-CNN model training process.

**Figure 4:** Misclassification examples: (a, b) false negatives; (c, d) false positives.

**Figure 5:** Colorectal lesion localization and classification using Mask R-CNN.

**Figure 6:** Our computer-aided diagnosis system workflow.

**Table 1:** Performance of different networks on test dataset.

Network	Accuracy (%)	Sensitivity (%)	Specificity (%)
AlexNet	85.5	78.9	92.2
VGG19	89.5	85.9	93.0
ResNet18	87.9	84.4	91.4
ResNet50	93.0	90.6	95.6
GoogLeNet	87.9	82.8	93.0

**Table 2:** Performance of Mask R-CNN model on test dataset.

Network	AP	AP_50_	AP_75_	AP_S_	AP_M_	AP_L_	AR	AR_10_	AR_100_	AR_S_	AR_M_	AR_L_
Mask R-CNN	67.6	90.3	83.3	100	65.1	64.8	75.4	78.2	78.2	100	79.9	76.5

## Data Availability

The data used to support the findings of this study are available from the corresponding author upon request.
